The article "A Novel Missense Variant in the Gene PPP2R5D Causes a Rare Neurodevelopmental Disorder with Increased Phenotype" was retracted in 2023. Reasons: signs of a paper mill; compromised peer review; unreliable results or conclusions.

# A Novel Missense Variant in the Gene *PPP2R5D* Causes a Rare Neurodevelopmental Disorder with Increased Phenotype

**DOI:** 10.1155/2021/6661860

**Published:** 2021-02-11

**Authors:** Lulu Yan, Ru Shen, Zongfu Cao, Chunxiao Han, Yuxin Zhang, Yingwen Liu, Xiangchun Yang, Min Xie, Haibo Li

**Affiliations:** ^1^The Central Laboratory of Birth Defects Prevention and Control, Ningbo Women and Children's Hospital, Ningbo, Zhejiang 315012, China; ^2^Department of Laboratory Medicine of Kunming Children's Hospital, Key Laboratory of Child Critical Disease Research of Yunnan Province, Kunming, Yunnan 650034, China; ^3^National Centre for Human Genetic Resource, National Research Institute for Family Planning, Beijing 100081, China

## Abstract

PPP2R5D-related neurodevelopmental disorder, which is mainly caused by de novo missense variants in the *PPP2R5D* gene, is a rare autosomal dominant genetic disorder with about 100 patients and a total of thirteen pathogenic variants known to exist globally so far. Here, we present a 24-month-old Chinese boy with developmental delay and other common clinical characteristics of PPP2R5D-related neurodevelopmental disorder including hypotonia, macrocephaly, intellectual disability, speech impairment, and behavioral abnormality. Trio-whole exome sequencing (WES) and Sanger sequencing were performed to identify the causal gene variant. The pathogenicity of the variant was evaluated using bioinformatics tools. We identified a novel pathogenic variant in the *PPP2R5D* gene (c.620G>T, p.Trp207Leu). The variant is located in the variant hotspot region of this gene and is predicted to cause PPP2R5D protein dysfunction due to an increase in local hydrophobicity and unstable three-dimensional structure. We report a novel pathogenic variant of *PPP2R5D* associated with PPP2R5D-related neurodevelopmental disorder from a Chinese family. Our findings expanded the phenotypic and mutational spectrum of PPP2R5D-related neurodevelopmental disorder.

## 1. Introduction

Neurodevelopmental disorders (NDDs) are a group of neurological diseases including intellectual disability (ID), autism spectrum disorders (ASDs), and language disorders with common clinical presentations that can affect cognitive, social, and motor abilities [1, 2]. NDDs have a strong genetic component, but the specific genetic factors underlying these disorders are heterogeneous and remain undefined for a large proportion of affected individuals [3]. With the development of sequencing techniques, numerous pathogenic genes have been identified in patients with NDDs [4]. Recently, whole exome sequencing (WES) has evolved as an effective strategy to discover and characterize causal variants for a significant portion of NDD patients [5].

PPP2R5D is a member of the phosphatase-2A (PP2A) family of phosphatases with critical roles in development, including maintaining neurons and regulating neuronal signaling. The *PPP2R5D* gene is located at chromosome 6p21.1, encoding the B56*δ* regulatory subunit of PP2A, an intracellular serine/threonine phosphatase. Variants in *PPP2R5D* are associated with mild to severe global developmental delay, hypotonia, ID, ASD, and behavioral abnormalities. Among these, pronounced hypotonia with delay in gross motor skills is the most frequently occurring symptom of PPP2R5D-related neurodevelopmental disorder [6–9]. Ever since PPP2R5D-related NDD was identified by Del-Mazo in 1996, more than 100 individuals with PPP2R5D-related NDD have been described. The disorder has a relatively limited mutational spectrum with thirteen pathogenic variants reported so far [10]. Here, we report a novel pathogenic variant in exon 5 of the *PPP2R5D* gene (c.620G>T, p.Trp207Leu) identified through trio-WES in a Chinese patient who presented hypotonia, macrocephaly, intellectual disability, speech impairment, and behavioral abnormalities. Meanwhile, some new significant clinical phenotypes possibly related to the *PPP2R5D* variants were also found.

## 2. Materials and Methods

### 2.1. The Patient General Information and Ethics Statement

Ethical approvals for the study were obtained from the Ningbo Women and Children's Hospital. Clinical information and blood specimens were obtained from the proband and related family members. The proband underwent thorough examination, including the physical growth and the behavior development assessment, MRI examination, laboratory examination, and EEG measurement. Written informed consent was provided by the proband's parents. The proband was born to nonconsanguineous parents after an uncomplicated pregnancy and delivery. Both parents of Chinese origin and the proband's brother were unaffected and healthy. There was no history of any neurodevelopmental abnormality in the family. The pedigree chart of his family is shown in Figure 1(a). The proband showed mild developmental delay (developmental quotient was 69.71), hypotonia, macrocephaly (head occipital frontal circumference was 47 cm > 2SD), prominent forehead, and open mouth at 10 months of age (Figures 1(b) and 1(c)). He also had a rash because of an allergy to egg whites, milk, and crabs (Figures 1(d)–1(f)). All routine laboratory tests revealed normal findings, including those of blood routine examination, serum biochemical indices, and amino acid metabolic levels. The electroencephalograms were normal. Magnetic resonance imaging (MRI) revealed dysgenesis of the corpus callosum, a reduction in brain parenchyma, widening of the cerebral sulci and fissures, and enlargement of the ventricular system at 10 months of age. The cerebral structures improved visibly when reexamined at 24 months of age (Figures 1(g)–1(l)). Other symptoms included delayed walking, speech impairment, and behavioral issues such as tantrums and trouble adjusting to new situations. The proband began speaking “mom” and “dad” at the age of 22 months and walking at the age of 23 months after rehabilitation.

### 2.2. DNA Extraction and Whole Exome Sequencing

Genomic DNA was extracted from peripheral blood leukocytes with informed consent and hospital ethical approval, using a QIAamp DNA Blood Mini Kit (Qiagen, Valencia, CA, USA), according to the manufacturer's protocol. DNA samples from the proband and his parents were subjected to WES using a HiSeq 2500 sequencing platform (Illumina, San Diego, CA, USA). The low-quality reads were filtered out from all sequencing data using a quality score 20 (Q20); the filtered sequencing data were compared to the human reference genome (hg19) using BWA. Then, variants were called by GATK and annotated to public databases by Annovar. The minor allele frequencies (MAFs) of all known variants were also reported according to their presence in the dbSNP 1000 Genomes Project (1000 GP), Exome Aggregation Consortium, and Exome Variant Server databases. Databases such as OMIM, ClinVar, HGMD, and SwissVar were used to determine mutation harmfulness and pathogenicity where appropriate. All whole-exome variants were subjected to biological effect analysis, which included the use of programs such as SIFT, MutationTaster, PolyPhen-2, PROVEAN, Human Splicing Finder, and MaxEntScan to predict whether an amino acid substitution or indel has an important biological effect. Variants were selected after combining the clinical information and then classified as pathogenic, likely pathogenic, variant of uncertain significance, likely benign, or benign according to the American College of Medical Genetics and Genomics (ACMG) guidelines.

### 2.3. Validating by Sanger Sequencing

To validate the variant screened by WES, Sanger sequencing was performed for the proband and family members. Genomic DNA was amplified by PCR using the PCR primers (forward, 5′-TGTCCTCTTTGACTTCGTG-3′; reverse, 5′-TTCTTGGCTATGTTTGGC-3′), which were designed with Primer 5 software. PCR conditions were as follows: 94°C for 10 min of initial denaturation followed by 30 cycles of amplification of 30 s at 94°C, 30 s at 60°C, and 45 s at 72°C. After reacting with BigDye Terminator v3.1, the PCR products were run on an ABI 3500DX Genetic Analyzer (Applied Biosystems, Foster City, CA) and analyzed by Sequencing Analysis Software 6. After validating the variant, family segregation was performed for all individuals.

### 2.4. Bioinformatics Analysis and Pathogenicity Assessment

The PPP2R5D protein sequence was obtained from the NCBI Protein Database (https://www.ncbi.nlm.nih.gov/protein/) in FASTA format. Online tools PolyPhen-2, SIFT, MutationTaster, and PROVEAN were used to predict the pathogenicity of the missense variant. Multiple sequence alignment and conservative analyses were performed using MEGA software. The hydrophobic properties of wild-type and mutant PPP2R5D protein were analyzed by ProtScale (https://web.expasy.org/protscale/). The 3D structures of wild-type and mutant protein were generated using the I-TASSER online server and PyMOL tool (http://zhanglab.ccmb.med.umich.edu/I-TASSER/, http://www.pymol.org/). The variant pathogenicity was assessed in standards and guidelines recommended by the American College of Medical Genetics and Genomics and the Association for Molecular Pathology (ACMG/AMP) [11].

## 3. Results

Trio-WES revealed 13 variants (Table 1) after filtering, among which *PPP2R5D* carried a de novo heterozygous variant (c.620G>T/p. Trp207Leu) (Figure 2(a)). The variant is located at a known variant hotspot (p. Trp207) within the B56 domain of this protein. The tryptophan at position 207 was highly conserved in different species (Figure 2(b)). By ProtScale analysis, it was found that the hydrophobicity of the protein increased because of the altered amino acid. Therefore, the change of this amino acid could generate alterations in the protein structure (Figure 2(c)). Furthermore, according to the I-TASSER tool prediction, there was a significant difference in the tertiary structural features between the wild-type and mutant PPP2R5D proteins. The Trp207Leu substitution impacted the formation of hydrogen bonds. Trp207 interacted with the Glu204 and Gln211 residues through hydrogen bonds, whereas the more hydrophobic residue leucine resulted in altered hydrogen bonding with Glu204 and Gln211 (Figures 3(a) and 3(b)). The amino acid replacement is not observed in unaffected family members and is absent from control databases, as well as 200 local controls. The majority of variant pathogenicity prediction tools supported the disease-causing consequence of this novel missense variant including a REVEL score of 0.7979. The variant is classified as pathogenic following the ACMG/AMP guidelines (PS2, PM1, PM2, PM5, PP2, and PP3) [8].

## 4. Discussion

PPP2R5D-related NDD is a recently characterized disorder. It is also known as Jordan's syndrome, named after Jordan Lang, the first child diagnosed in the United States. Since then, more than 100 cases have been identified across the globe [10]. The clinical manifestations of individuals with *PPP2R5D* variants included developmental delay and/or intellectual disability (100%), macrocephaly (78.26%), hypotonia (73.91%), ophthalmologic abnormalities (38.89%), and seizures (26.09%) [12].

To the best of our knowledge, only two Chinese patients with macrocephaly and NDDs have been reported with the same heterozygous missense variant (c.G592>A) of the *PPP2R5D* gene [13]. We reported a third Chinese patient with a novel pathogenic variant c.620G>T (p.Trp207Leu). Both two Chinese patients diagnosed previously had similar phenotypes comparable to other patients with *PPP2R5D* variants, including moderate global developmental delay, mild ID, frontal bossing, hypertelorism, and a history of epilepsy [13]. Some phenotypes of our patient are highly consistent with other PPP2R5D-related NDD patients, such as the specific feature of macrocephaly, prominent forehead, hypotonia, delayed speech and language development, and mild ID. In terms of nonspecific brain MRI results, the overall brain development of our patient was slower than that of other children of the same age. In addition to the aforementioned clinical manifestations, our patient also exhibited a serious allergic rash of the skin, which has not been described in previous cases. It is not clear whether this clinical manifestation is part of the symptomatology of PPP2R5D-related NDD, and it could possibly represent a new clinical phenotype.

PP2A complex is a heterodimeric core enzyme, which is composed of a scaffolding subunit A, a regulatory subunit B, and a catalytic subunit C [14]. B56*δ* is one of the isoforms of subunit B and is highly expressed in the human brain [15]. There is evidence that PP2A-PPP2R5D holoenzyme is involved in controlling the activity of the PI3K/AKT signaling pathway that plays a role in the maintenance and functioning of neurons [8]. According to the previous report, all ID-associated *PPP2R5D* variants except Pro53Ser resulted in deficient holoenzyme formation, most likely through a dominant-negative mechanism [7].

To date, a limited variant spectrum of *PPP2R5D* involving 12 missense variants and 1 nonsense variant has been identified (https://www.ncbi.nlm.nih.gov/clinvar/), and most of the *PPP2R5D* variants are located in exon 5 (Figure 2(d)). Among these variants, the Trp207Arg pathogenic variant is positioned in a conserved acidic loop of the PPP2R5D subunit critical for PP2A-PPP2R5D holoenzyme formation. The patient with the Trp207Arg variant learned to walk at the age of 2. In addition to moderate ID, developmental delay, hypotonia, and macrocephaly, he(she) also had scoliosis, hip dysplasia, and fatigue [7]. In the present study, a de novo missense variant c.620G>T (p.Trp207Leu) in exon 5 of the *PPP2R5D* gene was successfully identified in a Chinese patient with PPP2R5D-related NDD. The Trp207 amino acid in PPP2R5D is highly conserved among 10 species based on sequence alignment. Analyses by all the variant pathogenicity prediction tools supported the disease-causing consequence of this novel missense variant. In addition, the Trp207Leu substitution impacts the formation of hydrogen bonds of the Trp207 with the Glu204 and Gln211 residues and is predicted to increase the local hydrophobicity and disrupt the PPP2R5D protein structure/function. We therefore concluded that the Trp207Leu variant in PPP2R5D was the genetic etiology underlying PPP2R5D-related NDD in the proband. The research by Houge et al. [7] demonstrated deficient holoenzyme formation of PP2A due to decreased association of the mutant PPP2R5D subunit to the subunit A or subunit C. The Trp207Leu variant in the *PPP2R5D* gene may similarly perturb interactions between subunits of the PP2A complex [16]. Further functional studies will be focused on this rare variant site for deeper understanding of its functional implications.

In conclusion, a de novo *PPP2R5D* variant was identified in a Chinese patient with NDD through WES, which expanded the mutational and phenotypic spectrum of PPP2R5D-related NDD. There are no known effective treatments for NDDs associated with *PPP2R5D* variants. However, early intervention and rehabilitation therapy are available, which helped our patient to regain some impaired abilities. Further studies are required to assess the impact of *PPP2R5D* variants on neuronal functions and to facilitate the development of novel therapeutic strategies.

## Figures and Tables

**Figure 1:** A Chinese boy presents NDD. (a) Family pedigree. Arrow indicates the proband (II2); squares indicate males; circles indicate females; the filled symbol indicates the affected individual. (b–f) Facial and skin features of the patient at 10/19 months of age. (b, c) The patient displays macrocephaly, prominent forehead, and open mouth. (d–f) Allergic rash. Mainly concentrated on the limbs and trunk. (g–l) Brain MRI of the proband. (g–i) MRI showed a hypoplastic corpus callosum, temporal lobe parenchymal atrophy, enlargement of the ventricular system, and retardation of myelination of the white matter. (j–l) The bilateral temporal cortex was clear and plump (red arrows).

**Figure 2:** Identification of a missense variant in the *PPP2R5D* gene. (a) The novel heterozygous variant c.620G>T (p.Trp207Leu) in *PPP2R5D* was verified by Sanger sequencing. The variant is marked by a red arrow. (b) Protein alignment shows that the 207th tryptophan (marked by a red arrow) is highly conserved among different species. (c) Hydrophobicity of PPP2R5D protein. The prediction by ProtScale indicates an increase of local hydrophobicity around the site of p.Trp207Leu variant. WT: wild type. (d) The schematic diagram showing the gene structure of PPP2R5D. The variant in PPP2R5D occurs in exon 5, which causes G to T substitution at nucleotide 620 (NM_006245.3). Previously reported pathogenic variants are marked in black, and the variant identified in this study is highlighted in red.

**Figure 3:** Structural modeling of PPP2R5D protein. The I-TASSER tool predicts the structural changes caused by the p.Trp207Leu variant. (a) Amino acid at position 207 of wild-type PPP2R5D protein interacted with the Glu204 and Gln211 residues through hydrogen bonds which are presented as yellow dashed lines. (b) The formation of hydrogen bonds is predictably altered by the substitution of tryptophan by leucine at position 207.

**Table 1:** 13 variants in whole exome sequencing that were remaining after bioinformatic filtering.

Gene	Inheritance	Transcript	Exon/intron	Nucleotide alteration	Amino acid alteration	Chromosome position	Type	Disease's name (OMIM)	Proband	Father	Mother
PPP2R5D	[1]/[2]AD	NM_006245.3	Exon5	c.620G>T	p.W207L	chr6:429 75031	Nonsynonymous SNV	Mental retardation, autosomal dominant 35	Het	/	/
CREBBP	[1]/[2]AD	NM_004380.2	Exon31	c.6746_6757 del	p.R2249_Q2 252del	chr16:3778291-3778302:GCTGC TGCATGC:-	Nonframeshift deletion	Menke-Hennekam syndrome 1; Rubinstein-Taybi syndrome 1	Het	Het	/
PROKR2	[1]AD	NM_144773.3	Exon3	c.889G>A	p.V297I	chr20:5282952:C:T	Nonsynonymous SNV	Hypogonadotropic hypogonadism 3 with or without anosmia	Het	Het	/
UBA5	[1]AR	NM_024818.4	Exon11	c.1076G>A	p.G359D	chr3:132394712: G:A	Nonsynonymous SNV	Spinocerebellar ataxia, autosomal recessive 24; epileptic encephalopathy, early infantile, 44	Het	/	Het
YME1L1	1]AR [2]AR	NM_139312.2	Exon5	c.551A>T	p.H184L	chr10:27431366: T:A	Nonsynonymous SNV	Optic atrophy 11	Het	Het	/
NBAS	[1]AR [2]AR	NM_015909.3	Exon34	c.3938C>T	p.P1313L	chr2:15493828:G: A	Nonsynonymous SNV	Infantile liver failure syndrome 2; short stature, optic nerve atrophy, and Pelger-Huet anomaly	Het	Het	/
ARL13B	[1]AR	NM_182896.2	Exon2	c.106G>A	p.A36T	chr3:93714764:G:A	Nonsynonymous SNV	Joubert syndrome 8	Het	Het	/
ANK3	[1]AR	NM_020987.4	Exon37	c.6832A>C	p.K2278Q	chr10:61833807:T:G	Nonsynonymous SNV	Mental retardation, autosomal recessive, 37	Het	Het	/
MCEE	[1]AR	NM_032601.3	Exon2	c.275G>A	p.G92E	chr2:71351439:C:T	Nonsynonymous SNV	Methylmalonyl-CoA epimerase deficiency	Het	/	Het
UPB1	[1]AR	NM_016327.2	Exon2	c.142T>C	p.S48P	chr22:24896112:T:C	Nonsynonymous SNV	Beta-ureidopropionase deficiency	Het	Het	/
COL3A1	[1]AD [2]AR	NM_000090.3	Exon21	c.1472G>A	p.R491Q	chr2:189859788:G:A	Nonsynonymous SNV	Ehlers-Danlos syndrome, vascular type; polymicrogyria with or without vascular-type EDS	Het	/	Het
WFS1	[1]AD [2]AD [3]AR [4]AD [5]AD	NM_006005.3	Exon4	c.400G>A	p.A134T	chr4:6290798:G: A	Nonsynonymous SNV	Cataract 41; deafness, autosomal dominant 6/14/38; Wolfram syndrome 1; Wolfram-like syndrome, 54,46,autosomal dominant; diabetes mellitus, noninsulin-dependent, association with	Het	Het	/
ESCO2	[1]AR [2]AR	NM_001017420.2	Exon3	c.694C>T	p.R232C	chr8:27634519:C:T	Nonsynonymous SNV	Roberts syndrome; SC phocomelia syndrome	Het	/	Het

AD: autosomal dominant; AR: autosomal recessive; Het: heterozygous; Hom: homozygous; SNV: single nucleotide variants.

## Data Availability

The data used to support the findings of this study are included within the article.
